# Effect of Oxytocin Combined with Different Volume of Water Sac in High-Risk Term Pregnancies

This article has been retracted.

**DOI:** 10.1155/2022/1004816

**Published:** 2022-07-06

**Authors:** Hanna Mi, Na Sun

**Affiliations:** Department of Gynaecology and Obstetrics, People's Hospital of Putuo District, Zhoushan, Zhejiang, China

## Abstract

**Objective:**

The study estimated the impacts of water sac of different capacities combined with oxytocin (OXT) on pregnant women with high-risk term pregnancies.

**Methods:**

Women with high-risk term pregnancies who received OXT were enrolled to perform labor induction using 30  mL (group A), 80 mL (group B), and 150  mL (group C), followed by the comparisons regarding to the success rate of labor induction, cesarean section rate, duration of induced labor to labor, duration of the first stage of labor, postpartum blood loss, the incidence of adverse reactions, and the assessment of cervical ripening using Bishop Score. Besides, neonatal weight, Apgar score, as well as psychological status, and satisfaction of patients were compared among these groups.

**Results:**

As compared with group A, the success rate of induced labor was higher in groups B and C with lower cesarean section rate and shorter duration of induced labor to labor, but the duration of the first stage of labor in group B was the shortest among the three groups. The amount of postpartum hemorrhage decreased stepwise from groups A to B to C. In addition, groups A and B showed a reduced incidence of adverse reactions than group C, but the highest level of cervical ripening and highest patient satisfaction was revealed in group C and group B, respectively. Furthermore, the highest patient satisfaction was found in group B.

**Conclusion:**

The usage of an 80  mL water sac combined with OXT  in high-risk term pregnancy has ideal induction effects, which can guarantee maternal cervical maturity and shorten the time of the first stage of labor.

## 1. Introduction

Pregnant women suffer from various acute and chronic diseases and pregnancies, as well as adverse environmental and social factors, which can lead to fetal death, intrauterine growth retardation, congenital malformation, premature birth, neonatal diseases, and so on that constitute a high-risk pregnancy process called high-risk pregnancy [1]. In recent years, high-risk pregnancy has become increasingly common in the clinic, accounting for 8–12% of all pregnancies, an approximately four-fold increase compared to 2010 [2]. High-risk pregnancy not only poses a great threat to the newborn but may also lead to maternal death due to shock and massive hemorrhage during delivery [3]. Therefore, in clinic, it is necessary to focus on monitoring and additional targeted treatment for such pregnant women, so as to ensure maternal and child safety.

In clinical practice, induced uterine contractions are often used to help the fetus escape from the adverse intrauterine environment and reduce the occurrence of adverse pregnancy outcomes [4]. For normal pregnant women, labor can be induced by a variety of methods like low-dose oxytocin (OXT), prostate inhibitors, mifepristone, and pulse therapy [5]. However, due to the limitations of their own diseases, the only drug for induction of high-risk pregnant women is low-dose OXT—a therapy that can play a role in uterine contractions but has no significant effect on cervical dilation [6,7]. Therefore, there is an urgent need to find a more effective way to provide more effective protection for such pregnant women.

Water sac is an emerging technology in recent years, which can promote the softening and maturity of the cervix [8]. The placement of a water sac in the internal opening of the cervix can help artificially peel off the placenta and mechanically compress the cervix [9]. At present, some studies believe that water sac induction is safe for women with high-risk pregnancy, and it is expected to be a breakthrough to solve the problem of induced labor in high-risk pregnancy [10,11]. However, some other evidence has pointed out that the use of water sac may disrupt the normal state of the cervix of the mother [12]. Due to the current lack of authoritative and unified application guides, the use of water sac in high-risk pregnancies remains controversial.

This study compares the impacts of water sac of different capacities combined with OXT on postpartum cervical status of high-risk term pregnant women, aiming at providing more effective protection for maternal and child life safety and providing a more comprehensive reference for the subsequent application of water-sac induction of labor.

## 2. Data and Methods

### 2.1. Research Subjects

A total of 165 cases of high-risk term pregnancies who visited our hospital between January 2019 and March 2020 were selected as the research subjects for retrospective analysis. Among them, 54 cases were induced by 30 mL water sac (group A), 61 cases by 80 mL (group B), and 50 cases by 150 mL (group C). This study was carried out in strict accordance with the Declaration of Helsinki, and all the research subjects provided informed consent.

### 2.2. Eligibility Criteria

Patients who were in line with the diagnostic criteria of high-risk pregnancy [13] and water-sac-induced labor indications [14] with singleton pregnancy and fetal presentation were enrolled. In contrast, pregnant women with premature rupture of membranes, vaginitis, liver and kidney dysfunction, or fetal cardiac distress that need to stop pregnancy immediately were ruled out.

### 2.3. Treatment

All pregnant women received routine examinations, including B-ultrasound and fetal heart monitoring. At the same time, low-dose OXT (H34022979, An' hui Hongye Pharmaceutical Co., Ltd., China) was given as follows to induce labor. Day 1: OXT 2.5U was added into 500 mL of 0.5% glucose injection and then intravenously dripped. The infusion rate was appropriately adjusted according to the pregnant women's contractions to keep the contractions effective. Day 2: the parturient with a Bishop Score (BS) less than 6, which indicated an unripe cervix of patients [15], was given an OXT drip (same dose as day 1). Day 3: pregnant women with BS > 6 were subjected to artificial rupture of membranes, and those with BS < 6 were given OXT (same as day 1). No delivery after 3 days meant failure of induced labor and cesarean section was used instead. On this basis, patients in groups A, B, and C were induced by 30, 80, and 150 mL water sac, respectively, with the procedures as follows. First, in a lithotomy position, the vulva of the pregnant woman was routinely disinfected. The cervix was then exposed and disinfected with iodophor cotton balls. The front end of the water sac was inserted into the cervical canal, and 30, 80, or 150 mL of normal saline was injected slowly. The tail end of the water sac tube was ensured to be above the internal cervical orifice and the catheter was fixed on the inner thigh. After placing the water sac, the fetal heart and pregnant women's symptoms as well as the maternal physical symptoms were closely observed. The water sac was removed 20 h later and an artificial rupture of membranes was performed based on the BS score of the parturient.

### 2.4. Determination of Labor Induction Efficacy

Regular contractions lasting more than 30 seconds within 12 hours after treatment with the BS score increased by > 3 points were considered as remarkably effective. Effective was indicated if there were no regular contractions after treatment until the removal of the water sac for a period of time, with the BS score increased by 1–3 points. No regular contractions posttreatment nor changes or increase in the BS score was deemed ineffective. The induction success rate of induced labor = (remarkably effective + effective) cases/total cases × 100%. Moreover, the duration of induced labor to labor, the duration of the first stage of labor, the postpartum hemorrhage amount, and the cesarean section rate were recorded. BS results were recorded before (T0), and 2 h (T1) and 12 h induced labor (T2), as well as 2 h postpartum (T3).

### 2.5. Evaluation of Neonatal Status

Neonatal status was assessed via newborn weight, as well as using the Apgar Score (AS) [16] at 1 min and 5 min after birth, with the score positively associated with the neonatal status.

### 2.6. Assessment of Mental State

Before and after delivery, the maternal psychological state was evaluated by Self-rating Depression/Anxiety Scale (SDS/SAS) [17,18]. The standard cut-off is 50 points, with 50–59, 60–69, and *>* 69 being mild, moderate, and severe anxiety, respectively.

### 2.7. Determination of Adverse Reactions and Patient Satisfaction

The incidence of adverse reactions (ARs) was recorded between the application of the water sac for labor induction and at discharge. Patient satisfaction was assessed with the self-made nursing questionnaire (10-point scale), with 10, 7–9, 4–6, and 1–3 points being very satisfied, satisfied, need improvement, and dissatisfied, respectively. Satisfaction = (very satisfied + satisfied) cases/total cases × 100%.

### 2.8. Statistical Methods

SPSS22.0 software (SPSS, Inc., Chicago, IL, USA) was used for statistical analysis, and differences with *P* < 0.05 were considered significant. The measurement (mean ± SD) and enumeration data (*n* (%)) were analyzed via one-way analysis of variance (ANOVA) followed by Tukey's honest significant difference (HSD) and *χ*^2^ test, respectively.

## 3. Results

### 3.1. Comparison of Clinical Baseline Data

As shown in Table 1, comparisons among the three groups were conducted on baseline data regarding age, body mass index (BMI), gestational weeks, family history of disease, primipara, and household register, with no statistically significant differences (all *P* > 0.05)

### 3.2. Comparison of the Delivery Situation in High-Risk Term Pregnancies among the Three Groups

The effect of labor induction was compared, and the results are shown in Table 2. We found a similar success rate of labor induction in group B (80.33%) and group C (82.00%) (*P* > 0.05), higher than that of group A (61.11%) (*P* < 0.05). Similarly, the cesarean section rate differed significantly between group B (19.67%) and group C (18.00%) (*P* > 0.05), which was lower when compared to group A (38.89%) (*P* < 0.05). By comparing the delivery situation of the three groups (Figure 1), we found that there was no difference in the duration of induced labor to labor between groups B and C (*P* > 0.05), shorter than that of group A (*P* < 0.05). The duration of the first stage of labor was the shortest in group B (5.19 ± 1.65 h) among the three groups, followed by group A and group C (*P* < 0.05). The amount of postpartum hemorrhage decreased stepwise from groups A to B to C (*P* < 0.05).

### 3.3. Comparison of Maternal Cervical Status among the Three Groups

The results of BS scores before and after induced labor in the three groups are shown in Table 3. The three groups showed no difference in BS scores at T0 and T3 (*P* < 0.05), while at T1, the BS score was similar in groups B and C (*P* < 0.05), higher compared with group A (*P* < 0.05). At T2, the BS scores of the three groups from low to high were group A, group B, and group C (*P* < 0.05). In all the three groups, the BS score was the lowest at T0, increased continuously from T1 to T2, and reached the highest at T3 (*P* < 0.05).

### 3.4. Comparison of Neonatal Status among the Three Groups

No neonatal asphyxia or physiological defects occurred in the three groups, nor were there any notable differences among the three groups in neonatal weight and Apgar scores at 1 min and 5 min after birth (*P* < 0.05, Figure 2)

### 3.5. Comparison of Maternal Mental State among the Three Groups

SAS and SDS score results are detailed in Figure 3. The two scores differed insignificantly among the three groups before and after childbirth (*P* > 0.05) and were lower after childbirth compared with those before delivery (*P* < 0.05).

### 3.6. Comparison of ARs and Patient Satisfaction among the Three Groups

The statistics of ARs (Table 4) revealed no obvious difference in the incidence of ARs between groups A and B (*P* > 0.05), lower than that in group C (18.00%) (*P* < 0.05). Finally, the nursing satisfaction was surveyed and the results are presented in Table 5. The nursing satisfaction was 91.80% in group B, higher than that of groups A and C (*P* < 0.05).

## 4. Discussion

At present, induction of labor for pregnant women in the third trimester has become a common means in obstetrics and gynecology [19]. Among them, high-risk women are more worthy of labor induction in full-term pregnancy due to their various functional obstacles, so as to ensure the life safety of mothers and newborns [20]. In previous studies, we have found that low-dose OXT combined with water sac can increase the vaginal delivery rate of term pregnant women [21], but its application in high-risk pregnant women is still rare. As an emerging technique for inducing labor in recent years, water sac was reported to achieve the synthesis and to release the local endogenous prostaglandins in the cervix by dilating the cervix, thereby realizing labor induction [22]. Because of high safety, water sacs are favored by obstetrics and gynecology [23]. However, at present, there is still a great controversy in the selection of water sac capacity, so this study has important reference significance for the future clinical application of water sac.

Herein, we compared the delivery status of 3 groups of high-risk pregnancies using 30, 80, and 150 mL water sac, respectively. First, we can see that groups B and C had better induced labor effects and lower cesarean section rate than group A, indicating that 80 and 150 mL water sacs have better induced labor effects for high-risk pregnant women, being consistent with the research results of Delaney et al. [24]. Second, less duration of induced labor to labor was determined in groups B and C than in group A, which once again emphasizes better effects of 80 and 150 mL water sac. However, we found that the duration of the first stage of labor and postpartum hemorrhage volume in group C were the highest among the three groups, with an obviously higher incidence of ARs, suggesting low safety of the 150 mL water sac in high-risk pregnancy. As we all know, the mechanical stimulation of the water sac to the maternal cervix can react on the pituitary gland, induce OXT secretion, and accelerate patients' uterine contractions [22]. Therefore, we speculate that the difference among the three groups may be due to the small size of the 30 mL water sac that has weak stimulation on the maternal cervical canal, so the cervical maturity of the parturient is low and the effect of induced labor is not good. The 150 mL water sac, as the one with the largest capacity used in this study, has the strongest stimulation to the cervical canal, which can promote the cervical maturation faster and shorten the time of induced labor. But on the other hand, too big a water sac may bring greater pain to the maternal, which is not conducive to the subsequent delivery. Besides, the large capacity of the water sac can induce great mechanical damage to the parturient and easily cause complications such as cervical laceration, which leads to intensified pain in the parturient in the first stage of labor, as well as maternal hormone disorders that affect the regular contractions of the parturient, resulting in the prolongation of the first stage of labor [25]. Moreover, as the 150 mL water sac is placed in a high position of the uterus, it may move during maternal exercise, resulting in increased cervical compression and consequently leading to cervical laceration, umbilical cord prolapse, and other complications. Therefore, the safety of the 150 mL water sac is worse than that of the other two kinds. Then, we compared the BS scores of three groups of parturient during delivery, which also clearly showed the fastest cervical maturity in group C after the application of water sac, and the reason may be consistent with our above inference. The 80 mL water sac can effectively induce labor in high-risk pregnancies with a higher safety profile, so we believe that such a water sac has higher applicability.

In addition, postpartum depression, as a high-incidence mental illness of pregnant women after delivery, also seriously affects the health of mothers, their family members, and newborns [26,27]. Therefore, monitoring changes in mental state before and after childbirth is also one of the key items in obstetrics and gynecology at present [28]. The comparison of SAS and SDS scores among the three groups showed no difference, which once again emphasized the positive significance of water-sac-induced labor in high-risk pregnancies. Likewise, the comparison results of the neonatal situation revealed little difference among water sacs of the three sizes, indicating that they all have a relatively reliable guarantee for the safety of newborns. Finally, the survey results of nursing satisfaction show that group B has the highest satisfaction, which demonstrates that the 80 mL water sac is most suitable for high-risk pregnant women. The decrease in satisfaction in the other two groups, we hypothesize, may be due to the poor effect of induced labor in group A and the poor safety in group C.

Although this study analyzed the effect of water sacs with different capacities on induced labor in high-risk pregnancies, there are still many limitations to be improved. The number of cases included in this study was small, and the trial period was too short to evaluate the long-term prognosis of maternal and newborn babies. Second, we need to further compare the merits and demerits of water-sac induced labor with other labor induction methods, so as to provide a significance with more comprehensive reference opinions for the future clinical application of water-sac induced labor.

## 5. Conclusion

The usage of an 80 mL water sac combined with OXT in high-risk full-term pregnancy has ideal induction effects and high safety, which can effectively guarantee maternal cervical maturity and shorten the time of the first stage of labor, with high clinical popularization value.

## Figures and Tables

**Figure 1:** Comparison of the delivery situation in high-risk term pregnancies among the three groups. Note: patients were given low dose of oxytocin (OXT) combined with 30 mL (group A *n* = 54), 80 mL (group B *n* = 61), and 150 mL (group C *n* = 50) water sac. (a–c) Comparison of the duration of induced labor to labor (a), the duration of the first stage of labor (b), and the postpartum hemorrhage volume (c) among the three groups. ^*∗*^*P* < 0.05.

**Figure 2:** Comparison of neonatal status among the three groups. Note: patients were given low dose of oxytocin (OXT) combined with 30 mL (group A, *n* = 54), 80 mL (group B, *n* = 61), and 150 mL (group C, *n* = 50) water sac. (a, b) Comparison of the neonatal weight (a) and the Apgar scores (b) among the three groups.

**Figure 3:** Comparison of maternal mental state among the three groups. Note: patients were given low dose of oxytocin (OXT) combined with 30 mL (group A, *n* = 54), 80 mL (group B, *n* = 61), and 150 mL (group C, *n* = 50) water sac. (a, b) Comparison of the scores of the self-rating anxiety scale (SAS) (a) and self-rating depression scale (SDS) (b) among the three groups.

**Table 1:** Comparison of clinical baseline data among the three groups.

	Group A (*n* = 54)	Group B (*n* = 61)	Group C (*n* = 50)	*F* or *χ*^2^	*P*
Age	28.30 ± 3.31	27.90 ± 4.50	28.68 ± 4.11	0.515	0.598
BMI (kg/m^2^)	26.26 ± 2.54	25.79 ± 2.82	26.35 ± 2.57	0.502	0.606
Gestational weeks	39.67 ± 0.70	39.66 ± 0.89	39.36 ± 0.96	2.144	0.121
Family history of disease				0.431	0.806
Yes	8 (14.81)	10 (16.39)	6 (12.00)		
No	46 (85.19)	51 (83.61)	44 (88.00)		
Primipara				0.769	0.681
No	21 (38.89)	19 (31.15)	17 (34.00)		
Yes	33 (61.11)	42 (68.85)	33 (66.00)		
Household register				0.720	0.698
City	36 (66.67)	36 (59.02)	31 (62.00)		
Rural	18 (33.33)	25 (40.98)	19 (38.00)		

**Table 2:** Comparison of labor inducement effects.

Group	Remarkably effective	Effective	Ineffective	Induction success rate	Cesarean section rate
Group A (*n* = 54)	20 (37.04)	13 (24.07)	21 (38.89)	61.11%	38.89%
Group B (*n* = 61)	34 (55.74)	15 (24.59)	12 (19.67)	80.33%^*∗*^	19.67%^*∗*^
Group C (*n* = 50)	34 (68.00)	7 (14.00)	9 (18.00)	82.00%^*∗*^	18.00%^*∗*^
*χ* ^2^				7.675	
*P*				0.022	

Note: ^*∗*^ means *P* < 0.05 compared with group A.

**Table 3:** Changes of Bishop score during delivery in three groups of parturients.

Group	T0	T1	T2	T3	F	*P*
Group A (*n* = 54)	3.59 ± 1.06	6.15 ± 0.76 ^&^	7.54 ± 1.02 ^&@^	8.89 ± 0.86 ^&@%^	318.0	*<* 0.001
Group B (*n* = 61)	3.46 ± 1.13	6.70 ± 0.86^*∗*^^&^	7.97 ± 0.75^*∗*^^&@^	8.98 ± 0.81 ^&@%^	434.6	*<* 0.001
Group C (*n* = 50)	3.48 ± 1.25	6.72 ± 1.17^*∗*^^&^	8.32 ± 0.47^*∗*^^#&@^	9.12 ± 0.85 ^&@%^	323.2	*<* 0.001
F	0.207	6.531	12.920	0.988		
P	0.814	0.002	*<* 0.001	0.375		

Note: BS results were recorded before (T0), and 2 h (T1) and 12 h induced labor (T2), as well as 2 h postpartum (T3). ^*∗*^ means *P* < 0.05 compared with group A, # means *P* < 0.05 compared with group B, & means *P* < 0.05 compared with T0 in the same group, @ means *P* < 0.055 compared with T1 in the same group, and % means *P* < 0.05 compared with T2 in the same group.

**Table 4:** Incidence of maternal adverse reactions (ARs) in three groups.

	Umbilical cord shedding	Strong cervical contractions	Cervical tear	ARs
Group A (*n* = 54)	1 (1.85)	1 (1.85)	0 (0.0)	3.70%
Group B (*n* = 61)	2 (3.28)	1 (1.64)	1 (1.64)	6.56%
Group C (*n* = 50)	3 (6.00)	4 (8.00)	2 (4.00)	18.00%^*∗*^^#^
*χ*2				7.172
P				0.028

Note: ^*∗*^ means *P* < 0.05 compared with group A and ^#^ means *P* < 0.05 compared with group B.

**Table 5:** Nursing satisfaction of three groups of puerperae.

Group	Very satisfied	Satisfy	Needs improvement	Dissatisfied	Total satisfaction
Group A (*n* = 54)	24 (44.44)	18 (33.33)	6 (11.11)	6 (11.11)	77.78%
Group B (*n* = 61)	39 (63.93)	17 (28.87)	4 (6.56)	1 (1.64)	91.80%^*∗*^
Group C (*n* = 50)	20 (40.00)	17 (34.00)	7 (14.00)	6 (12.00)	74.00%^#^
*χ* ^2^					9.066
P					0.011

Note: ^*∗*^ means *P* < 0.05 compared with group A and ^#^ means *P* < 0.05 compared with group B.

## Data Availability

The data used to support the findings of this study are included within the article.
